# In-vitro antibiofilm activity of chlorhexidine digluconate on polylactide-based and collagen-based membranes

**DOI:** 10.1186/s12903-019-0979-y

**Published:** 2019-12-26

**Authors:** Jan-Luca Rudolf, Corina Moser, Anton Sculean, Sigrun Eick

**Affiliations:** 1 Department of Periodontology, School of Dental Medicine, University of Bern, Bern, Switzerland; 2 Department of Restorative, Preventive and Pediatric Dentistry, School of Dental Medicine, University of Bern, Bern, Switzerland

**Keywords:** Guided tissue regeneration, Bioresorbable membrane, Antiseptic, Bacterial colonization, Periodontal ligament fibroblasts, Gingival epithelial cells

## Abstract

**Background:**

In Guided Tissue Regeneration (GTR), barrier membranes are used to allow selective cell populations to multiply and to promote periodontal regeneration. A frequent complication is membrane exposure to the oral cavity followed by bacterial colonization. The purpose of this in-vitro-study was to elucidate, if rinsing with a chlorhexidine digluconate solution (CHX) prevents bacterial adhesion, and whether it interferes with attachment of periodontal ligament (PDL) fibroblasts and epithelial cells to membrane surfaces.

**Methods:**

Firstly, two bioresorbable membranes (polylactide-based and collagen-based) were dipped into 0.06% CHX and 0.12% CHX, before biofilms (2-species representing periodontal health, 6-species representing a periodontitis) were formed for 2 h and 8 h. Subsequently, colony forming units (cfu) were counted. Secondly, the membranes were treated with CHX and inoculated in bacteria suspension two-time per day for 3 d before cfu were determined. In additional series, the influence of CHX and bacterial lysates on attachment of epithelial cells and PDL fibroblasts was determined. Parameter-free tests were applied for statistical analysis.

**Results:**

Cfu in “healthy” biofilms did not differ between the two membranes, more cfu were counted in “periodontitis” biofilm on collagen than on polylactide membranes. One-time dipping of membranes into CHX solutions did not markedly influence the cfu counts of both biofilms on polylactide membrane; those on collagen-based membrane were significantly reduced with being 0.12% CHX more active than 0.06% CHX. More-fold CHX dipping of membranes reduced concentration-dependent the cfu counts of both biofilms on both membranes. In general, the number of attached gingival epithelial cells and PDL fibroblasts was higher on collagen than on polylactide membrane. Lysates of the periodontopathogenic bacteria inhibited attachment of PDL fibroblasts to membranes. CHX decreased in a concentration-dependend manner the number of attached gingival epithelial cells and PDL fibroblasts.

**Conclusions:**

The present in-vitro results appear to indicate that membranes in GTR should only be used when bacteria being associated with periodontal disease have been eliminated. An exposure of the membrane should be avoided. Rinsing with CHX may prevent or at least retard bacterial colonization on membrane exposed to the oral activity. However, a certain negative effect on wound healing cannot be excluded.

## Background

Guided Tissue Regeneration (GTR) is an established surgical technique in reconstructive periodontal surgery. Barrier membranes are used to mechanically isolate the treated defects in order to prevent proliferation of epithelial and connective tissue cells into the wound [1, 2]. Thus, they support proliferation of periodontal ligament and bone cells onto the root surfaces and into the defect which leads ultimately to formation of connective tissue attachment (i.e. new cementum with perpendicularly inserting collagen fibers) and bone [1, 2]. Resorbable membranes have been developed to avoid surgical removal of the membrane, thus minimizing the risk of damaging the newly formed tissues. Animal and human-derived collagen-based membranes and polyester-based membranes consisting of polylactic acid and its copolymers are routinely used in the clinical setting [1]. The membranes should not induce any inflammatory reaction and must present a degradation profile that matches with new tissue formation [1]. As recently reported in a systemic review, treatment of intrabony defects with GTR using collagen membranes results in a mean of 1.58 mm higher clinical attachment level gain compared with open flap debridement alone [3].

Complications which might occur after surgical procedure are exposure of the membrane, bacterial contamination and infection [4]. Exposure of a membrane is a frequently reported complication following regenerative periodontal surgery [5]. Following exposure to the oral cavity, bacterial colonization immediately occurs implying an increased risk of infection, thus jeopardizing the regeneration process and the final clinical outcomes [6–8].

Bacteria associated with periodontal disease may interfere with wound healing following GTR. If the oral cavity of a patient is colonized by these bacteria, the same species can be also found in high percentages at the sites, where surgery was performed [9]. It has been shown that bacteria attached to membranes inhibit the attachment of periodontal ligament fibroblasts [10]. In vitro bacteria adhere in high numbers to membranes, at which adhesion was significantly higher to collagen membranes compared to non-resorbable PTFE-based barriers [11].

In order to decrease the bacterial load, chlorhexidine digluconate solutions are usually applied post-surgically, but very rarely the effect of chlorhexidine on bacterial contamination of membranes was investigated. Chen et al. [10] found an inhibition of *Aggregatibacter actinomycetemcomitans* adhesion, but also a decreased viability of 50% of PDL fibroblasts in the presence of 0.0015% CHX. Clinically, the application of a CHX chip was beneficial in periodontal regeneration [12]. In another study, biofilm accumulation was followed in volunteers on removable membranes after rinsing with CHX solution for 4 h and 24 h. The results showed an inhibitory effect of CHX but also an influence of the membrane material [13]. In a similar experimental design, but with a follow-up of 4 weeks, no effect of CHX on preventing or retarding bacterial adhesion was seen [14].

The purpose of the present in-vitro-study was to investigate, if rinsing with a chlorhexidine digluconate solution (CHX) may prevent bacterial adhesion and biofilm formation on bioresorbable synthetic and collagen-based membranes using two different biofilms (i.e. one representing periodontal health and the other representing periodontal disease). Furthermore, the question was to be answered whether rinsing with a chlorhexidine digluconate solution, may interfere with the attachment of periodontal ligament (PDL) fibroblasts or epithelial cells to the membranes.

## Material and methods

### Membranes

Two bioresorbable membranes were included, one consisting of polylactide and blended with citric acid ester (GUIDOR® Bioresorbable Matrix Barrier; Sunstar Suisse SA; Etoy, Switzerland), and the other was a membrane consisting of porcine pericardium collagen (Jason®, kindly provided by botiss materials GmbH, Zossen, Germany).

From these membranes, test specimens with a size of 5 × 5 mm were prepared.

### Chlorhexidine digluconate solution

CHX without additives were obtained from the pharmacy of the University hospital Bern and prepared as a 0.12% (CHX0.12), 0.06% (CHX0.06), and 0.015% (CHX0.015) CHX.

### Microorganisms

The microorganisms *Streptococcus gordonii* ATCC 10558, *Actinomyces naeslundii* ATCC 12104, *Porphyromonas gingivalis* ATCC 33277, *Tannerella forsythia* ATCC 43037, *Fusobacterium nucleatum* ATCC 25586, and *Parvimonas micra* ATCC 33270. were included in the assays. *S. gordonii* and *A. naeslundii* represent early colonizers, whereas *P. gingivalis*, *T. forsythia*, *F. nucleatum* and *P. micra* are known to be clearly associated with periodontal diseases. Prior to the experiments, all strains were precultivated on Schaedler agar plates (Oxoid, Basingstoke, UK) with 5% sheep blood (JP. Mischler, Switzerland) overnight in an anaerobic atmosphere or with 5% CO_2_ (*S. gordonii* ATCC 10558). Bacteria concentration was adjusted to OD600 nm = 0.5 in 0.9% v/w NaCl (equivalent to 10^9^ bacteria/ml). Then mixed suspension was prepared by mixing 1 part *S. gordonii* with 2 parts *A. naeslundii* (and each 4 parts of the other species for six-species mixture).

### Cells

Human PDL fibroblasts were anonymously collected from periodontally healthy patients during regular orthodontic treatment following written informed consent. This procedure is approved by the Ethics Committee of the University of Bern. Human PDL fibroblasts were placed in T-25 cell culture flasks containing DMEM (Life Technologies / Invitrogen, Paisley, UK) with 10% foetal calf serum (FCS; Life Technologies / Invitrogen) to grow to confluency. At the starting of the experiments, the fibroblasts were always in the 4th – 6th passage.

The telomerase-inactivated gingival keratinocytes (TIGK) kindly provided by R. Lamont, University of Louisville, KY, USA [15]) were maintained in cell cultivation media (Keratinocyte Growth Medium, KGM-Gold, Lonza, Basel, Switzerland). Confluent monolayers of PDL fibroblasts and TIGK cells were detached by trypsin / EDTA and the amount of epithelial cells was adjusted to about 10^6^ / 1 ml of cell cultivation media.

### Biofilm formation on membranes

Two biofilms were used, one consisting of *S. gordonii* and *A. naeslundii* representing a biofilm associated with periodontal health (“healthy” biofilm), and another one consisting of all six species representing a periodontopathogenic biofilm (“periodontal” biofilm). Suspensions of the two or six bacterial strains were mixed with nutrient broth (Wilkins Chalgren broth + 5% sheep blood) in a ratio 1: 19. Then test specimens were dipped first into 25% serum (Sigma-Aldrich, Buchs, Switzerland) solution and thereafter into CHX0.12, or CHX0.06 for 1 min before placing into 24-well-plates, and exposing to the bacterial suspension. After an incubation time for 2 h and 8 h under anaerobic conditions, biofilms were removed from the surface. After mixing by pipetting, a serial dilution was made and the total cfu counts assessed. Further, in case of the six-species biofilms, the loads of *P. gingivalis* and *T. forsythia* were determined by using real-time PCR [16].

In a second series of experiments, membranes were treated as before, but after an incubation time of 8 h, membranes were exposed again to the respective chlorhexidine digluconate solution or 0.9 w/v NaCl (control) for 1 min. Then, the solution was removed and bacterial suspension was added again for 16 h. Thereafter, the procedure was repeated twice per day to simulate clinical rinsing of the oral cavity with chlorhexidine digluconate solution two-times per day. After three days, the bacterial counts were determined as described above.

### Adhesion of PDL fibroblasts and gingival epithelial cells (TIGK)

The membrane specimens were dipped into 25% serum solution and thereafter into chlorhexidine digluconate solution in three concentrations (CHX0.12, CHX0.06, CHX0.015 (to mimic a possible dilution gradient) or 0.9 w/v NaCl (control)) for 1 min. Afterwards, the specimens were placed in 24-well-plates and PDL fibroblasts or TIGK were added. Membranes were incubated with PDL fibroblasts with 5% CO_2_ for 72 h or with TIGK for 24 h (each about 10^5^ cells / mm^2^), before the numbers of adherent fibroblasts were counted.

### Influence of microorganisms on adhesion of PDL fibroblasts and TIGK

Experiments with PDL fibroblasts and TIGK cells were repeated in the presence of bacterial lysates. Bacterial suspensions of two or six species were prepared as described before and adjusted to the concentrations 10^7^ / ml, 10^8^ / ml, and 10^9^ /ml. Then the suspensions had been exposed to ultrasonication of 160 W for 10 min, and filtered through membranes with a pore size of 400 μm. The through-flow or 0.9% w/v NaCl was finally added to the cell culture medium in a ratio 1: 9.

Finally, one concentration of bacteria (10^7^/ml) and chlorhexidine digluconate solution (CHX0.015) were selected to study a potential interference of both components. Treatment of barrier membranes and the other processing steps were made as described above.

### Expression of IL-8 and TGFβ1 in PDL fibroblasts

Moreover, the potential effects of CHX and bacterial lysates on PDL fibroblasts, which are critical for gingival wound healing, were analyzed at gene expression level. Membranes were dipped before adding PDL fibroblasts into CHX0.015 or lysates of bacterial suspensions (10^8^ /ml) were added. After the treatment of cells, RNA was extracted by using the innuPREP RNA Mini Kit (Analytic Jena, Jena, Germany) and cDNA generated from 100 ng total RNA by using the GoScript™ Reverse Transcription System (Promega, Madison, WI, USA) according to the manufacturers’ instructions. Thereafter real-time PCR using GoTaq® qPCR Master Mix (Promega) with respective primers was used to quantify mRNA expression of IL-8 and TGFβ1. The primers for IL-8 (primer: fwd: 5′-CACTGCGCCAACACAGAAAT-3′, rev.: 5′-TGGCCCTTGGCCTCAATTTT-3′; # BC013615.1) and TGFβ1 (primer: fwd.: 5′-CCAGATCCTGTCCAAGCTGC-3′; rev.: 5′-GCTGAGGTATCGCCAGGAAT-3′; # NM_000660.6) were designed by using PRIMER-BLAST being a tool for finding specific primers (National Center for Biotechnology Information, U.S. National Library of Medicine, Bethseda, USA). GADPH [17] served as the reference gene.

### Statistical analysis

All experiments were performed in independent quadruplicates in at least two series. Statistical analyses based on log10 of bacterial counts (total colony forming units (CFU) and counts of selected periodontopathogens) as well as on the number of attached cells / mm^2^.

Parameter-free tests were applied for statistical analysis. After performing Kruskal-Wallis-H-test for comparing all groups, Mann-Whitney-U-test determined differences to the control each. Only for analyzing mRNA expression, Student t-test was used. The level of significance was set to *p* = 0.05. Software SPSS 24.0 (IBM SPSS Statistics, Chicago, IL, USA) was used.

## Results

### CHX before biofilm formation

Without exposing to CHX, in median 5.11 log10 cfu and 5.59 log10 cfu were counted in “healthy” biofilms on polylactide membrane after 2 h and 8 h, the respective number for the collagen membrane was 5.02 log10 after 2 h and 5.68 log10 cfu after 8 h. The differences between the two membranes were not statistically significant. CHX solutions did not remarkly influence the cfu counts on the polylactide membrane, cfu counts were reduced only by 0.09 log10 in median 8 h after dipping the membrane into CHX0.12 (Fig. 1a). On the collagen membrane, CHX0.06 and CHX0.12 reduced the cfu counts of the “healthy” biofilm by 1.13 log10 after 8 h of biofilm formation (each *p* = 0.001; Fig. 1b).

**Fig. 1:** Total cfu counts (**a**, **b**) of a 2-species “healthy” biofilm, and total cfu counts of a 6-species “periodontal” biofilm (**c**, **d** and counts of *Porphyromonas gingivalis* (**e**, **f**) and *Tannerella forsythia* (**g**, **h**) in “periodontal” biofilm after dipping initially polylactide (**a**, **c**, **e**, **g**) and collagen (**b**, **d**, **f**, **h**) membranes into 0.06 and 0.12% chlorhexidine digluconate solution (CHX0.06 and CHX0.12) and culturing the biofilms for 2 h and 8 h. Presented are median and 10, 25, 75 and 90 percentiles. *p < 0.05 vs. control. **p < 0.01 vs. control

Without exposing to CHX in median 5.01 log10 cfu and 5.70 log10 cfu were counted in “periodontal” biofilms on polylactide membrane after 2 h and 8 h, the respective number for the collagen membrane was 5.06 log10 after 2 h and 7.46 log10 cfu after 8 h. The difference between the two membranes was statistically significant at 8 h (*p* < 0.001). And there was also a statistically significant difference between “healthy” and “periodontal” biofilms on polylactide and collagen membranes each after 8 h (*p* = 0.016; *p* = 0.004). CHX did not remarkly influence the cfu counts on the polylactide membrane (Fig. 1c). On the collagen membrane, the CHX0.12 reduced the cfu counts of the “periodontal” biofilm by 2.22 log10 and by 2.66 log10 cfu when membranes were exposed initially to CHX0.06 and CHX0.12 (each *p* = 0.001; Fig. 1d).

Determination of selected periodontopathogens by real-time PCR counts not only bacteria being able to form colony forming units. The numbers include also metabolically inactive and in part dead bacteria. Following, the results are not totally comparable to those obtained by culturing. Within the “periodontal” biofilms and without CHX exposure, counts of *P. gingivalis* and *T. forsythia* were higher on the collagen membrane than on the polylactide one at 8 h (*p* < 0.001; *p* = 0.001). CHX did influence neither the *P. gingivalis* counts nor the *T. forsythia* counts on the polylactide membrane (Fig. 1e, g). On the collagen membrane, less *P. gingivalis* were counted after exposing membrane to CHX (CHX0.06, CHX0.12 both p < 0.001) at 8 h of biofilm formation (Fig. 1f). Also less *T. forsythia* were counted after exposing the collagen membrane to CHX (CHX0.06 *p* = 0.006, CHX0.12 *p* < 0.001) at 8 h of biofilm formation (Fig. 1h).

### More-fold CHX rinsing in biofilm formation

Without exposing to CHX, in median 7.28 log10 cfu were counted in “healthy” biofilms on polylactide membrane at 3 d, the respective number for the collagen membrane was 7.56 log10. The difference between the two membranes was statistically significant (*p* = 0.038). CHX0.06 and CHX 0.12 reduced the cfu counts by 3.52 log10 and 5.97 log10 (each *p* < 0.001) on the polylactide membrane (Fig. 2a). On the collagen membrane (Fig. 2b), the decrease was 4.05 log10 cfu (CHX0.06; *p* < 0.001) and 6.26 log10 cfu (CHX0.12; p < 0.001).

**Fig. 2:** Total cfu counts (**a**, **b**) of a 2-species “healthy” biofilm, and total cfu counts of a 6-species “periodontal” biofilm (**c**, **d** and counts of *Porphyromonas gingivalis* (**e**, **f**) and *Tannerella forsythia* (**g**, **h**) in “periodontal” biofilm after more-fold dipping of polylactide (**a**, **c**, **e**, **g**) and collagen (**b**, **d**, **f**, **h**) membranes into 0.06 and 0.12% chlorhexidine digluconate solution (CHX0.06 and CHX0.12) and culturing biofilms for 3 d. Presented are median and 10, 25, 75 and 90 percentiles. **p < 0.01 vs. control

Without exposing the membrane to CHX in median 7.24 log10 cfu were counted in “periodontal” biofilms on polylactide membrane at 3 d, the respective number for the collagen membrane was 7.53 log10. The difference between the two membranes was statistically significant (*p* = 0.001). However, there was no difference of total bacterial counts between the “healthy” biofilm and the “periodontal” biofilm neither on polylactide nor on collagen membranes. CHX0.06 reduced the cfu counts of “periodontal” biofilms by 2.86 log10 on the polylactide (Fig. 2c) and by 4.28 on the collagen (Fig. 2d) membranes (each *p* < 0.001). After morefold applying CHX 0.12 in median no cfu was counted on both membranes.

Within the “periodontal” biofilms and without CHX exposure, counts of *P. gingivalis* and *T. forsythia* were higher on the collagen membrane than on the polylactide membrane at 3 d (*p* = 0.015; *p* = 0.021). CHX0.06 and CHX0.12 reduced the *P. gingivalis* counts on polylactide (Fig. 2e) and collagen (Fig. 2f) membranes (each *p* < 0.001). CHX0.12 also reduced *T. forsythia* counts on the polylactide membrane (*p* = 0.001; Fig. 2g). On the collagen membrane, both CHX were active against *T. forsythia* (each *p* < 0.001; Fig. 2h).

### Adhesion of PDL fibroblasts and TIGK

Without exposing to CHX in median 16.5 PDL fibroblasts / mm^2^ were counted on the polylactide membrane after 3 d, the respective number for the collagen membrane was 63.0 PDL fibroblasts / mm^2^. The difference between the two membranes was statistically significant (*p* < 0.001). Applying CHX0.015 to the polylactide membrane did not change the number of attached PDL fibroblasts, but CHX0.06 and CHX0.12 reduced these numbers on membranes (*p* = 0.004, *p* = 0.005; Fig. 3a). On collagen membranes, there was a decrease of attached cells after applying any CHX vs. control (each p < 0.001; Fig. 3b).

**Fig. 3:** Attached PDL fibroblasts (**a**, **b**; after 72 h of incubation) and TIGK (**c**, **d**; after 24 h of incubation) to polylactide (**a**, **c**) and collagen (**b**, **d**) membranes after dipping initially membranes into 0.015, 0.06 and 0.12% chlorhexidine digluconate solution (CHX0.015, CHX0.06 and CHX0.12; **a**, **c**). Presented are median and 10, 25, 75 and 90 percentiles. **p < 0.01 vs. control

Without exposing to CHX, in median 15.5 TIGK cells / mm^2^ were counted on the polylactide membrane after 24 h, the respective number for the collagen membrane was 89.0 cells / mm^2^. The difference between the two membranes was statistically significant (*p* < 0.001). Applying CHX initially to membranes did not change statistically significantly the number of attached TIGK cells on polylactid membranes (Fig. 3c). On collagen membrane, there was a decrease of attached cells vs. control after applying any CHX (p < 0.001; Fig. 3d).

#### Lysates of microorganisms and adhesion of PDL fibroblasts and gingival epithelial cells to membranes

Lysates of the two bacterial species being associated with periodontal health did not change attachment of PDL fibroblasts to the polylactide membrane (Fig. 5a). On the collagen membrane, there were more attached PDL fibroblasts in part (lysates from 10^7^ bacteria/ml: *p* = 0.021 and 10^8^ bacteria/ml: p < 0.001). However, when combined with CHX0.015, the number of attached PDL fibroblasts decreased when compared to control (*p* < 0.001; Fig. 4b).

**Fig. 4:** Attached PDL fibroblasts (**a**, **b**, **c**, **d**; after 72 h of incubation) and TIGK (**e**, **f**, **g**, **h**; after 24 h of incubation) to polylactide (**a**, **c**, **e**, **g**) and collagen (**b**, **d**, **f**, **h**) membranes in the presence bacterial lysates (prepared from two species being associated with periodontal health (**a**, **b**, **e**, **f**) or six species associated with periodontal disease (**c**, **d**, **g**, **h**) in three concentrations and in part after dipping initially membranes into 0.015% digluconate solution (CHX) *p < 0.05 vs. control. Presented are median and 10, 25, 75 and 90 percentiles. **p < 0.01 vs. control

Lysates of the six bacterial species being associated with periodontal disease decreased further the low number of attached PDL fibroblasts to the polylactide membrane (lysates from 10^8^ bacteria/ml: *p* = 0.039 and 10^9^ bacteria/ml: *p* = 0.004; Fig. 4c). On the collagen membrane, there were also less attached PDL fibroblasts when lysates from 10^9^ bacteria/ml were added (*p* = 0.032; Fig. 4d). When bacterial lysates were added to membranes dipped before into CHX0.015; the number of attached PDL fibroblasts was lower when compared to control (polylactide membrane: *p* = 0.003, collagen membrane: p = 0.004).

Lysates of the two bacterial species being associated with periodontal health and lysates of the six bacterial species being associated with periodontal disease did not change attachment of TIGK to the polylactide membrane (Fig. 4e; g). On collagen, both lysates decreased the number of attached TIGK cells (*p* = 0.031 – *p* < 0.001; Fig. 4f, h).

When bacterial lysates were added to the collagen membrane dipped before into CHX0.015; the numbers of attached TIGK cells were lower when compared to control (2-species: p < 0.001, 6-species: *p* = 0.018).

### Expression of IL-8 and TGFβ1 in PDL fibroblasts

Due to the low number of attached PDL fibroblasts on the polylactide membrane, amount of extracted RNA was insufficient to determine expression of cytokines. Following, only results on collagen membrane can be presented. CHX0.015 provoked an increase of IL-8 expression in PDL fibroblasts (*p* = 0.014). There was also a tendency to higher expression of IL-8 in the presence of bacterial lysates of “periodontal biofilm” without reaching statistical significance (*p* = 0.062). TGFβ1-expression did not differ significantly between membranes with and without exposure to CHX0.015 or bacterial lysates (Fig. 5).

**Fig. 5:** mRNA expression of IL-8 (**a**) and TGFβ1 (**b**) of PDL fibroblasts on collagen membranes after dipping into 0.15% CHX solution and in the presence of bacterial lysates being associated with periodontal health and periodontal disease. Presented are means and SD related to expression on collagen membranes without CHX and bacterial lysates. *p < 0.05 vs. control

## Discussion

The present in-vitro study has evaluated the effect of chlorhexidine digluconate on bacterial contamination and adhesion of epithelial cells and PDL fibroblasts to two commercially available membranes. The results revealed an inhibition of bacterial adhesion to membranes by chlorhexidine digluconate. However, there were also clear differences between the two membranes, not only regarding the activity of chlorhexidine, but also regarding the attachment of host cells and bacterial biofilm formation.

Three major types of membranes are commercially available, non resorbable (PTFE-based, or e-PTFE-based), resorbable tissue-derived collagen membranes and resorbable polyester (polyglycolic acid, polylactid acid, poly-ε-caprolactone) membranes [18]. In vitro studies have shown a higher bacterial adhesion on collagen membrane than on e-PTFE- and PTFE- based membranes [11], or glycolide fiber membrane [19]. The limited attachment on the polyester membrane is discussed in the light of a hydrophobicity of the material [19]. Our results confirm the higher bacterial adhesion on collagen-based membrane when compared with polylactide-based membrane but only when a bacterial mixture consisting of periodontopathogens was used. Bacterial species being associated with periodontal health colonized the polylactide membrane and the collagen membrane similarily.

One of the main functions of GTR membranes is to inhibit epithelial down-growth. In particular, if the membrane is exposed to the oral cavity an epithelial seal may prevent colonization of bacteria at the deeper parts of the membranes. The GTR membrane should function also as a substrate for the migration of cells for wound healing and regeneration [20]. Not only bacteria, but also the oral epithelial cells and periodontal ligament fibroblasts should preferably attach to the membrane. Previous studies have confirmed the preference of host cells to collagen membrane thus resulting in better adhesion of PDL fibroblasts than on glycolide fiber membrane [21] and ePTFE-membrane [10, 21].

In the present study, released compounds of bacteria being associated with periodontal health did not negatively influence attachment of PDL fibroblasts to membranes. In contrast, there was a negative influence of products by bacteria being associated with periodontal disease. Bacteria being associated with periodontal disease use collagen as a nutrient source [22, 23] and moreover it was shown that proteolytic enzymes of *P. gingivalis* can degrade collagen membranes [24]. But also a cleavage of host cell receptors on membranes and of cell adhesion molecules enabling the contact between the cells can be suggested. E.g., *P. gingivalis* proteases affect cell adhesion capability of fibronectin and tenascin C to fibroblasts [25] and they are able to degrade adhesion molecules essential for epithelial integrity [26].

In a clinical study the presence of *P. gingivalis* at the time-point of surgery was found to be negatively associated with the outcome, the attachment gain was 1.5 mm less when compared with no presence [9]. This underlines the need to eliminate or at least to reduce periodontopathogenic bacteria before regenerative periodontal surgery using membranes.

This in-vitro study mimicked an exposure of the membrane to the oral cavity which happens quite frequently after periodontal surgery. Data from the literature report a frequency of 44% [27] up to 87% [28]. The high frequency of membrane exposure and the resulting problem of bacterial colonization underline the need to search for options to inhibit biofilm formation on membranes. One possibility is the modification of the membrane itself. Loading of an electrospun poly(ɛ-caprolactone)-gelatin nanofiber membrane with metronidazole showed favourable results in vitro and in animal model [29]. In vitro, also the addition of amoxicillin or tetracycline inhibited the adhesion of *A. actinomycetemcomitans* or *Streptococcus mutans* [19]. Further, silver nanoparticles incorporated in a membrane inhibited adhesion of periodontopathogenic bacteria [30]. However, the available clinical studies report different outcomes. A collagen membrane with added metronidazole did not show a superiority to a membrane without [31]. Using a membrane loaded with 25% doxycycline resulting in more probing depth reduction than using one without antibiotic [32].

The second approach is the adjunctive application of antimicrobials, either topically or systemically. Regarding the systemic use of antimicrobials, the data are very limited. A study applying minocycline before surgery and thereafter amoxicillin and doxycycline has failed to show any benefit by the antibiotics [33]. At present, rinsing with chlorhexidine digluconate two-times per day is recommended after GTR surgery [4].

In the present study the additional application of CHX was investigated. The starting point were two commonly used CHX concentrations in the mouthrinses, 0.06 and 0.12%. No commercially available product was included. However, it cannot be excluded that additives in the CHX formulations may interfere with its activity [34].

The first experiments mimicked a one-time exposure of the membrane to CHX. This may simulate a clinical situation at the time of surgery. The initial dipping into CHX decreased bacterial counts and those of *P. gingivalis* and *T. forsythia* on the collagen membrane, the anti-adhesive activity was higher when CHX0.12 was was used in comparison with CHX0.06. The colonization of the polylactide membrane was not influenced by dipping into any CHX solution. Chlorhexidine digluconate is a cationic molecules which is attaching to negatively charged surfaces [35], when attached it has a high substantivity [36] meaning a long lasting post-antimicrobial activity. Further, the collagen membrane is hydrophilic [19] and the polylactide membrane is rather hydrophobic [37], which may play a role both in bacterial adhesion as well as in the attachment of CHX.

The second series of experiments mimicked the clinical situation of membrane exposure where CHX is applied twice per day. The dipping of the membranes two-times per day for three days decreased remarkably bacterial colonization of both bacterial species being associated with periodontal health and of those being associated with periodontal disease. Again the antiadhesive activity was higher on the collagen membrane than on polylactide membrane, but in contrast to the one-time dipping a reduction of the bacterial adhesion was seen on both membranes.

Also the effect of the CHX on adhesion of PDL fibroblasts and gingival epithelial cells was investigated. A lower concentration than the commercially ones was included as it can be expected that the concentration of chlorhexidine is lowered in deeper regions when contacting the membrane. Dipping the collagen membrane in this low concentrated CHX (0.015%) already decreased the numbers of attached PDL fibroblasts and increased expression of the pro-inflammatory cytokine IL-8. The negative effect of CHX on the attachment of PDL fibroblasts and epithelial cells on collagen membrane was concentration dependent. Meanwhile cytotoxicity of chlorhexidine was reported in many studies. Only short-time exposure of primary human fibroblasts to commercially available concentrations of chlorhexidine gluconate and digluconate affects extremely their viability [34, 38], in a scratching assay no defect closure was seen after 3 min of 0.002% chlorhexidine gluconate [38]. The inhibition of attachment of oral cells to membranes by CHX contradicts the positive effect in inihibiting bacterial adhesion and underlines that membranes should not be dipped into CHX before placement during surgery.

## Conclusions

In summary, the polylactide membrane may be a treatment option for patients who reject medical devices derived from animals. Bacterial colonization seems to be more limited compared to a collagen-based membrane. However, this obvious advantage has to be seen in contrast with the relatively low attachment of gingival epithelial cells and periodontal ligament fibroblasts.

The in-vitro results of this study suggest using membranes in guided tissue regeneration only when bacteria being associated with periodontal disease have been elimiated. An exposure of the membrane should be avoided. Rinsing with CHX may prevent or at least retard bacterial colonization on membranes being exposed in the oral activity. However, a certain negative effect on wound healing cannot be excluded.

## Data Availability

The datasets used and/or analyzed during the current study available from the corresponding author on reasonable request.

## Abbreviations

Cfu: Colony forming unit
CHX: Chlorhexidine digluconate solution(s)
CHX0.015: 0.015% chlorhexidine digluconate solution
CHX0.06: 0.06% chlorhexidine digluconate solution
CHX0.12: 0.12% chlorhexidine digluconate solution
GTR: Guided tissue regeneration
IL-8: Interleukin-8
PDL: Periodontal ligament
TGF-β1: Transforming growth factor β1
TIGK: Telomerase-inactivated gingival keratinocytes
